The article "Identification of Cigarette Smoking-Related Novel Biomarkers in Lung Adenocarcinoma" was retracted in 2024. Reasons: signs of a paper mill; suspected computer-generated content; unreliable results or conclusions; concerns about the data.

# Identification of Cigarette Smoking-Related Novel Biomarkers in Lung Adenocarcinoma

**DOI:** 10.1155/2022/9170722

**Published:** 2022-06-19

**Authors:** Yuan Zhang, Qiong Wang, Ting Zhu, Hui Chen

**Affiliations:** ^1^Department of Respiratory Medicine, Zhenhai Hospital of Traditional Chinese Medicine, Ningbo, 315000 Zhejiang, China; ^2^Department of Preventive Medicine of Traditional Chinese medicine, Jiangnan Hospital Affiliated to Zhejiang Chinese Medical University (Hangzhou Xiaoshan Hospital of Traditional Chinese Medicine), Hangzhou 310000, Zhejiang, China

## Abstract

**Objective:**

The aims of this study were to screen the gene mutations that are able to predict the risk of cigarette smoking-related lung adenocarcinoma (LUAD) and to evaluate its prognostic significance.

**Methods:**

Clinical data and genetic information were retrieved from the TCGA database, and the patients with LUAD were divided into three groups including never smoking, light smoking, and heavy smoking according to cigarette smoking dose. Differentially mutated genes (DMGs) of each group were analyzed. At the same time, the function of DMGs in three smoking groups was evaluated by GO function and KEGG pathway analysis. The driver genes and protein variation effect of DMGs were performed to further screen key genes. The survival characteristics of the gene expression and mutation of those genes were analyzed and plotted to visualize by the Kaplan-Meier model.

**Result:**

The DMGs for different smoking doses were identified. The driver and deleterious mutation in the DMGs were screened and gene interaction network was constructed. The DMGs with driver mutations and deleterious mutations that were associated with the overall survival in the heavy smoking patients were considered as the candidate genes for novel markers of smoking-related LUAD. The final novel risk factor gene was identified as MYH7 and the high express of MYH7 in LUAD correlation with patients' gender, lymph node metastasis, T stage, and clinical stage.

**Conclusions:**

In summary, it can be concluded that MYH7 is a novel biomarker for heavy smoking-related LUAD and it is significantly correlated with the prognosis of lung cancer and is related to the clinical characteristics of lung cancer.

## 1. Introduction

Lung cancer is the most common malignancy in humans which leads to high cancer-related deaths worldwide. Lung adenocarcinoma (LUAD) is the main histological type, including more than 40% of lung cancer [1, 2]. The 5-year survival rate of patients with LUAD is less than 10%, and 90% of them die of complications related to tumor metastasis [3, 4]. Most patients with LUAD are diagnosed at advanced stages, thus miss best opportunities for surgical treatments. To make matters worse, LUAD is not sensitive to radiotherapy and chemotherapy, and the prognosis of patients with LUAD remains poor. In recent years, the incidence and mortality of lung cancer have been increasing year by year, which has caused serious negative effects on patients and society [5]. Many studies have shown that cigarette smoking is the main cause of lung cancer [6–8]. Tobacco smoke contains polycyclic aromatic hydrocarbons and the nicotine-derived nitrosamines, which induce gene mutations in known oncogenes such as *KRAS* and *TP53* [9]. Moreover, it is reported that tobacco aldehydes inhibit the DNA repair [10]. Smoking increases the risk for development of the lung cancer via these mechanisms, and thus, smoking-associated LUAD has its specific gene mutations compared with general LUAD. In the current context of precision treatment of cancer, it is necessary to explore biomarkers or molecular targets for cigarette smoking-associated LUAD. Understanding the mechanism of the occurrence and development of cigarette smoking-associated LUAD contributes to identifying therapeutic targets and approaches for the prevention and management.

The article "Identification of Cigarette Smoking-Related Novel Biomarkers in Lung Adenocarcinoma" was retracted in 2024. Reasons: signs of a paper mill; suspected computer-generated content; unreliable results or conclusions; concerns about the data.

In this study, data of gene mutation for lung adenocarcinoma patients were downloaded from The Cancer Genome Atlas (TCGA), and the differentially mutated genes (DMGs) among three groups including never smoking, light smoking, and heavy smoking groups were screened. We analyzed the gene function enrichment of the specific DMGs for heavy smoking patients and identified the oncogenic drivers in them. We also analyzed gene-gene interaction of the specific DMGs and their association with prognosis for overall survival. Combining the above results, we found a novel biomarker, *MYH7*, with high occurrence of mutation in heavy smoking patients. There are to date few reports for *MYH7* in lung cancer. Therefore, *MYH7* can be used as a novel target for the diagnosis of smoking-associated lung cancer or for targeted precision therapy targeting *MYH7*.

## 2. Materials and Methods

### 2.1. Datasets

The clinical data and gene expression information of lung cancer patients were downloaded from the American Cancer Genome Atlas Database (TCGA), and lung adenocarcinoma (Broad, Cell 2012) dataset was used to obtain lung cancer patients' information. A total of 184 samples were included in this study. A total of 65,768 somatic mutations were detected.

### 2.2. Identification of Differentially Mutated Genes

Differentially mutated gene analysis for the never smoker, light smoker, and heavy smoker groups in the LUAD dataset was performed by using the clinical enrichment function of the maftools package in R software. *p* value < 0.05 was defined as the significant difference.

The article "Identification of Cigarette Smoking-Related Novel Biomarkers in Lung Adenocarcinoma" was retracted in 2024. Reasons: signs of a paper mill; suspected computer-generated content; unreliable results or conclusions; concerns about the data.

### 2.3. Functional Annotation

As for the obtained different genes, Gene Ontology (GO) and Kyoto Encyclopedia of Genes and Genomes (KEGG) pathway annotation were performed with the R package (clusterProfiler). GO annotation was carried out from the aspects of biological process (BP), molecular function (MF), and cellular component (CC). Fisher's test was used to calculate the *p* value of significance level, so as to screen the GO with significant enrichment of different genes. The *p* value < 0.01 was marked with red as the significant enrichment item and the blue as the nonsignificant item. KEGG database was used to explore the signal pathway of significantly differentially expressed gene enrichment, with *p* value < 0.05 as the threshold.

### 2.4. Driver Gene Analysis Based on Mutation Location Clustering

Oncogene mutations usually gather at specific locations of proteins (also known as mutation hot spots), and the mutations in these domains are beneficial to the growth or proliferation of cancer cells. We used OncodriveCLUST algorithm to cluster the mutation sites of gene bases to identify cancer genes. The key information calculated included the number of mutation hot spots, the number of mutations clustering in the hot spots, the length of amino acids corresponding to the protein, the proportion of clustering mutations in all mutations of the gene, and the *p* value and FDR values. The smaller the value, the stronger the driving force.

### 2.5. Mutation Damaging Was Assessed Based on PROVEAN and SIFT Software

Homologous proteins were found in the database, and protein sequences with high similarity and consistent function were selected for multisequence PSI-BLAST alignment to evaluate the conserved protein sites, and the risk was evaluated by PROVEAN/SIFT database score.

### 2.6. Interacting Network Analysis

The STRING database (https://string-db.org/) is used to explore the interactions between proteins and genes. The SRING database contains experimental data, direct interactions, and indirect functional correlations between proteins and obtains the PPI interaction network diagram.

### 2.7. Statistical Analysis

The gene expression information and overall survival (OS) data were obtained from TCGA database. The Kaplan-Meier analysis was used to calculate the hazard ratio (HR), and the survival curve was drawn. *p* < 0.05 was considered to be significantly related to the prognosis of lung cancer patients.

## 3. Results

### 3.1. Screening of Differential Mutation Genes in Lung Cancer Patients with Different Smoking Levels

The somatic gene mutation profiles and clinical data were acquired from the TCGA database, which included 184 patients. The result of the survival analysis showed that the smoking situation significantly associated with patient's OS (Table 1, *p* = 0.023). Lung adenocarcinoma patients were divided into nonsmoking group, light smoking group, and heavy smoking group based on their total amount of smoking (the product of the number of packs smoked and the number of years) up to the time of tumor diagnosis: heavy (>10), light (>0 and<10), and never (=0). The mutation status of patients in each group was statistically analyzed, and the results are shown in Figure 1. As can be seen from the figure, the single nucleotide missense mutation was the dominant mutation in the three types of patients with different smoking levels. Patients in the nonsmoking group mutated the base type to replace thymine cytosine nucleotide with cytosine nucleotide (C>T), followed by cytosine nucleotide substitution for adenine nucleotide substitution (C>A), while cytosine nucleotide substitution for adenine nucleotide substitution in light and heavy smoking groups (C>A) is the most common, followed by cytosine nucleotide instead of thymine (C>T). The top 10 mutant genes in the nonsmoking group were *EGFR*, *ZFHX3*, *CDC42BPA*, *TP53*, *SPHKAP*, *SLC17A6*, *Scand3*, *RelN*, *GRTN2A*, and *DIDO1*. The top 10 mutant genes in light smoking group were *TTN*, *MUC16*, *HMCN1*, *FLG*, *TP53*, *EGFR*, *USH2A*, *CSMD3*, *NALCN*, and *HSPG2*. The top 10 mutant genes in the heavy smoking group were *TTN*, *MUC16*, *LRP1B*, *CSMD3*, *RyR2*, *USH2A*, *TP53*, *SPTA1*, *ZFHX4*, and *KRAS*. The 1122 DMGs were identified in heavy smoking, 432 DMGs were identified in light smoking, and 327 DMGs were identified in never smoking, and the significant genes are shown in Figure 2.

The article "Identification of Cigarette Smoking-Related Novel Biomarkers in Lung Adenocarcinoma" was retracted in 2024. Reasons: signs of a paper mill; suspected computer-generated content; unreliable results or conclusions; concerns about the data.

### 3.2. GO and KEGG Pathway Analysis of Mutated Differential Genes

Using GO analysis, the difference of gene has been studied, and the results are shown in Figure 3; the difference of gene biological pathways is mainly related to cell adhesion, involving the main molecular function of the ion channels combining exercise, calcium ion, and extracellular matrix structure; these genes mainly located in the plasma membrane and organelle membrane, which are involved in cell information exchange, may be related to the spread of cancer cells to metastasize. KEGG pathway results are shown in Figure 3. These genes were significantly correlated with adhesion, ECM receptor interaction, olfaction transduction, and other signaling pathways.

### 3.3. Protein Variation Effect of Mutated Genes and Candidate Marker Genes

In order to validate the protein variation effect of mutation genes between never smoking, light smoking, and heavy smoking patients, boxplots of model genes were drawn, and both PROVEN and SIFT programs showed that the variation effect scores for the protein functions between never, light, and heavy smoking groups were significantly different (*p* < 0.05, Figure 4), while PROVEN and SIFT scores were conflicting in light smoking group. Mutations in light smokers were more deleterious in the SIFT scores while contrary in the PROVEN scores. Driver gene analysis was performed on the mutation data of lung cancer dataset based on mutation location clustering. The results of cancer driver genes with *p* value less than 0.05 are shown in Table 2. The oncogenes significantly associated with lung cancer were KRAS, NR4A2, CDKN2A, EGFR, OR5AS1, OR5D14, DOCK11, TFEB, and ZNF335.

Based on the results of differential mutation, cancer driving gene analysis, and mutation harmfulness analysis, the genes were intersected. Differential mutations that may be cancer drivers in the never smoker, light smoker, and heavy smoker groups were obtained (*p* value < 0.1), and damaging and deleterious genes are considered as key candidate genes in PROBEAN/SIFT prediction, which are arranged by mutation frequency, as shown in Table 2.

### 3.4. Interacting Networks of Important Differential Mutants

The interaction between proteins of cancer-driving genes was explored based on the STRING database, which included experimental data, results mined from PubMed abstracts and integrated data from other databases, as well as results predicted by bioinformatics methods. The PPI interaction network diagram is shown in Figure 5. It can be seen from the diagram that CDKN2A, KRAS, EGFR, TLR4, and TP53 with high-grade index are the core genes, followed by STK11, SPTA1, MYH8, MYH7, and MYO10, and most of the core genes have been reported. Literature mining was performed for searching the association of those genes to the smoking lung cancer. The results showed that only MYH7 and MYH8 genes had not been reported yet, and they were candidate genes related to lung cancer of new types of smoking. Although there is an enrichment of MYH7 mutation in heavy smoking patients, the mutation loci varied in the patients (Supplementary Table 1).

### 3.5. Novel Biomarkers of Smoking-Related LUAD

PubMed was used to search for papers related to the key node genes of result 2.4 and cancer caused by smoking. The results showed that only *MYH7* and *MYH8* genes had not been reported yet and were candidate genes related to lung cancer caused by heavy smoking. Survival curve analysis was conducted on these two genes using the prognosis data from lung adenocarcinoma (TCGA, provisional) database, and the results are shown in Figure 6. As can be seen from the figure, high expression of *MYH7* gene significantly reduced the prognostic survival rate of patients. The high expression of *MYH8* gene had no significant effect on the prognostic survival rate. Therefore, *MYH7* was screened as a new smoking-induced lung cancer target gene.

The article "Identification of Cigarette Smoking-Related Novel Biomarkers in Lung Adenocarcinoma" was retracted in 2024. Reasons: signs of a paper mill; suspected computer-generated content; unreliable results or conclusions; concerns about the data.

## 4. Discussion

In this study, we focused on the analysis of mutated genes associated with tobacco smoking in LUAD. We identified specific mutations in LUAD patients with heavy smoking that were distinct from the nonsmoking group. Among these mutations, we screened the genes with driver mutations and those with deleterious mutations. Considering that these mutated genes have regulatory relationships and affect the occurrence of LUAD through common pathways, we subsequently performed gene interaction analysis for these mutated genes and constructed a gene network for smoking-related LUAD centered on genes known to be high frequency mutated in LUAD, such as *KRAS* and *TP53*. Based on the results of the literature search, most of these smoking-related core genes (*CDKN2A*, *EGFR*, *KRAS*, *TLR4*, *TP53*, *SPTA1*, and *STK11*) we identified have been reported in many studies for their association with lung cancer. However, *MYH7* has not been studied to elaborate its association with lung cancer. In LUAD, *MYH7* has a high mutation frequency (11 of 90), so *MYH7* can be used as a novel diagnostic biomarker. Meanwhile, the gene expression of *MYH7* correlated with the overall survival of LUAD patients and the tumor stage and lymph node metastasis of patients, suggesting that *MYH7* is associated with the progression of LUAD, and thus precise targeted therapies targeting MYH7 can be carried out in the future.

Current research on *MYH7* has focused on studies in cardiomyopathies, as it is predominantly expressed in the normal human ventricle. Mutations in this gene are associated with familial hypertrophic cardiomyopathy, myosin storage myopathy, dilated cardiomyopathy, and Laing early-onset distal myopathy [11–14]. In our results, *MYH7* was shown to be highly expressed in LUAD tumor tissue. In addition, only a small number of studies have shown that *MYH7* is associated with tumorigenesis. Sun et al. reported that *MYH7* is one of the top ten hub genes in *PTEN* mutation prostate cancer [15]. Huang et al. reported that mutations in MYH7 occur in Epstein-Barr virus-associated intrahepatic cholangiocarcinoma [16]. This paper is the first to propose that the lack of function of *MYH7* is one of the causes of LUAD, especially for smoking-associated LUAD.

The article "Identification of Cigarette Smoking-Related Novel Biomarkers in Lung Adenocarcinoma" was retracted in 2024. Reasons: signs of a paper mill; suspected computer-generated content; unreliable results or conclusions; concerns about the data.

Although cigarette smoking is the main cause of lung cancer, the incidence of lung cancer is increasing among nonsmokers. It is estimated that about 25% of lung cancer cases are observed in nonsmokers, and some studies have observed that 40% of nonsmoking men and 31.2% of nonsmoking women have no known exposure history to major carcinogens [17, 18]. If lung cancer in nonsmokers were considered as a single cancer, it would be the seventh leading cancer death in the world [17]. If the current growth rate of nonsmoking lung cancer continues, it is predicted that nonsmoking lung cancer will be the main type of lung cancer in the next 10 years [19]. Current evidence shows that nonsmoking lung cancer shows a different pattern from smokers' lung cancer, and there are essential differences between nonsmoking lung cancer and smoking-related lung cancer in terms of gender, clinical characteristics, and molecular genetic changes [20, 21]. Heavy smokers were found to have many specific gene mutations in this study, while never smokers did not seem to have specific gene mutations, compared to other smoking patients. Therefore, the results of the present study cannot explain the etiology of non-smoking-related LUAD. Considering the high rate of non-smoking-related lung cancer as well, more studies are still needed for non-smoking-related LUAD, but we suggest that studies can be conducted at levels other than gene mutations.

## Figures and Tables

**Figure 1:** The profile of somatic mutations for never smokers (a), light smokers (b), and heavy smokers (c) in LUAD, respectively. From top to bottom, each row is the statistics of mutation types, the type and number of mutation bases (vertical axis is classified; horizontal axis scale is counted), and the count box diagram of mutation number and mutation species in each sample.

**Figure 2:** Genes with *p* value < 0.05 for differential mutation significance in a given group are shown, sorted from left to right by significance of difference in different subgroups. The horizontal axis shows the gene names, the vertical axis shows the proportion of mutations in different subgroups, and the bar chart colors show the subgroups, corresponding to the figure notes on the right.

**Figure 3:** GO and KEGG pathway enrichment analysis of differentially mutated genes.

**Figure 4:** The box chart showing the harmfulness of mutations in patients with different smoking conditions (harmless and neutral mutation data have been screened out). (a) The result predicted by the PROVEAN and (b) the result predicted by the SIFT.

**Figure 5:** Gene-gene interaction of specific DMGs in driver and deleterious mutations. The circular nodes represent genes and the straight lines represent the reciprocal relationships that exist in genes. The size of the node represents the degree value, and the color shade represents the *k*-core value size.

The article "Identification of Cigarette Smoking-Related Novel Biomarkers in Lung Adenocarcinoma" was retracted in 2024. Reasons: signs of a paper mill; suspected computer-generated content; unreliable results or conclusions; concerns about the data.

**Figure 6:** The association of *MYH7* mutation with overall survival (*p* = 0.24) (a) and the association of *MYH7* expression with overall survival (*p* = 0.02) (b) of LUAD patients and with the sample type (*p* = 0.001) (c), tumor stages (*p* = 0.004) (d), race (*p* = 0.02) (e), gender (*p* = 0.61) (f), nodal metastasis (*p* = 0.03) (g), and *TP53* mutation (*p* = 0.23) (h) in LUAD.

**Table 1:** Clinical characteristics of patients with different smoking degrees.

Clinical	Never smoker	Light smoker	Heavy smoker	*p* value
Smoking amount	0	1-10	11-128	
Age	67.59 (43-87)	59.25 (42-78)	65.69 (38-84)	0.205
Gender				0.015
Men	7	7	66	
Women	20	10	52	
TNM stage				0.567
I	16	13	60	
II	5	1	24	
III	4	3	15	
IV	1	0	8	
Overall survival (OS)	21.69	19.86	14.13	0.023

**Table 2:** Genes in driver and deleterious mutation obtained from the DMGs for different smoking conditions. Genes were arranged by mutation frequency.

Hugo_Symbol	Total mutated	Mutated samples	Hugo_Symbol	Total mutated	Mutated samples	Hugo_Symbol	Total mutated	Mutated samples
TP53	67	63	CNTNAP5	21	17	SCN11A	11	9
TTN	144	61	CTNND2	20	17	ARAP2	10	9
MUC16	95	51	KIF2B	20	17	MYO10	10	9
LRP1B	85	48	LRP2	20	17	OR10AG1	10	9
SPTA1	49	39	MYO18B	20	17	PCDHA9	10	9
ZFHX4	51	36	EPHA5	20	16	GABRA5	9	9
KRAS	36	36	SORCS3	18	15	OR4M2	9	9
PCLO	48	34	POTEC	16	15	WSCD1	11	8
XIRP2	47	34	KEAP1	15	15	THBS2	10	8
PCDH15	36	29	PCDH10	18	14	MKRN3	9	8
CSMD1	40	26	TRPS1	17	14	AGBL1	8	8
LPHN3	30	26	CMYA5	15	14	CDKN2A	8	8
RP1L1	31	25	LRRC4C	15	14	GP2	8	8
RELN	29	24	MYH7	15	14	OR5D14	8	8
DNAH9	34	23	CDH7	13	13	SLC6A2	8	8
EGFR	26	23	KCNT2	15	12	LPA	8	7
ZNF804A	26	22	KIAA1211	15	12	ADCY5	7	7
ZNF536	30	21	LRRTM4	13	12	OR5B17	7	7
CUBN	27	21	MYH8	14	11	PKP2	7	7
FAM5C	27	21	BRAF	12	11	SAGE1	7	7
STK11	21	21	FAM71B	12	11	TSHR	7	7
BAI3	24	20	TLR4	12	11	VSTM2A	7	7
MXRA5	22	20	CNTN5	11	11	ADAM21	7	6
TPTE	22	20	POM121L12	11	11	FCRLA	7	6
CDH10	24	19	TGIF2LX	11	11	OR5AS1	7	6
FLG2	21	18	SLC17A6	13	10	C7orf10	6	6
DNAH3	20	18	MMP16	12	10	CLCNKA	6	6
EPHA3	20	18	OR2M2	11	10	NR4A2	6	6
PRDM9	20	18	TRHDE	11	10	OR10A4	6	6
CSMD2	19	18	KCNJ3	10	10	OR10Z1	6	6
PKHD1L1	26	17	RAG1	10	10	TRIM48	6	6

## Data Availability

The data used to support the findings of this study are included within the article.

## Supplementary Materials

Supplementary Materials Supplementary Table 1: the mutated sites of MYH7 in the heavy smoking patients.
